RETRACTED

# Melatonin Attenuates Ischemia/Reperfusion-Induced Oxidative Stress by Activating Mitochondrial Fusion in Cardiomyocytes

**DOI:** 10.1155/2022/7105181

**Published:** 2022-01-10

**Authors:** Xiaoling Ma, Shengchi Wang, Hui Cheng, Haichun Ouyang, Xiaoning Ma

**Affiliations:** ^1^Department of Critical Care Medicine, Shijiazhuang People's Hospital, Shijiazhuang, Hebei 050000, China; ^2^Department of Cardiology, The Seventh Affiliated Hospital, Southern Medical University, China

## Abstract

Myocardial ischemia/reperfusion (I/R) injury can stimulate mitochondrial reactive oxygen species production. Optic atrophy 1- (OPA1-) induced mitochondrial fusion is an endogenous antioxidative mechanism that preserves the mitochondrial function. In our study, we investigated whether melatonin augments OPA1-dependent mitochondrial fusion and thus maintains redox balance during myocardial I/R injury. In hypoxia/reoxygenation- (H/R-) treated H9C2 cardiomyocytes, melatonin treatment upregulated OPA1 mRNA and protein expression, thereby enhancing mitochondrial fusion. Melatonin also suppressed apoptosis in H/R-treated cardiomyocytes, as evidenced by increased cell viability, diminished caspase-3 activity, and reduced Troponin T secretion; however, silencing *OPA1* abolished these effects. H/R treatment augmented mitochondrial ROS production and repressed antioxidative molecule levels, while melatonin reversed these changes in an OPA1-dependent manner. Melatonin also inhibited mitochondrial permeability transition pore opening and maintained the mitochondrial membrane potential, but *OPA1* silencing prevented these outcomes. These results illustrate that melatonin administration alleviates cardiomyocyte I/R injury by activating OPA1-induced mitochondrial fusion and inhibiting mitochondrial oxidative stress.

## 1. Introduction

Timely myocardial reperfusion with thrombolysis can effectively save the viable heart muscle and limit the myocardial infarction area [1]. However, myocardial ischemia/reperfusion (I/R) injury and cell death often occur in the process of reperfusion; although, this concept has only recently become widely accepted. There are four major manifestations of myocardial I/R injury: (1) reperfusion-induced ventricular arrhythmia; (2) myocardial stunning, a type of systolic dysfunction that occurs when oxidative stress and endoplasmic reticulum calcium imbalance impairs cardiomyocyte contractile elements; (3) microvascular obstruction, the inability to reperfuse the ischemic site due to capillary injury, impaired vasodilation, external capillary compression caused by myocardial swelling, microembolism caused by arteriosclerotic plaque fragments, platelet microthrombosis, soluble vasomotor, thrombogenic substance release, and neutrophil blockage; and (4) fatal myocardial reperfusion injury, the death of viable cardiomyocytes due to redox imbalance, abnormal calcium signal, and mitochondrial malfunction [2–7]. The first two manifestations of myocardial I/R injury are reversible, while the latter two are irreversible and lack effective therapeutic approaches.

RETRACTED

Mitochondria may be damaged during myocardial I/R injury, and mitochondrial damage has been identified as a primary cause of reactive oxygen species (ROS) overproduction [8–10]. Mitochondrial fusion is a protective mechanism that both repairs damaged mitochondria and improves the stability of the mitochondrial DNA by fusing poorly structured mitochondria with the network of healthy mitochondria [11–13]. Mitochondrial fusion has been reported to be reduced during myocardial I/R injury; thus, many clinical protective tools have been created to enhance mitochondrial fusion and inhibit mitochondrial ROS overload [14–16].

Melatonin is an endogenous hormone with potential cardioprotective effects. Melatonin administration has been found to sustain mitochondrial function and thus reduce a variety of cardiovascular disorders, such as diabetic cardiomyopathy, myocardial I/R injury, septic cardiomyopathy, cardiac remodeling, and vital myocarditis [17–19]. However, the action of melatonin on mitochondrial fusion is not fully understood. Therefore, our experiments were used to determine whether melatonin mediates cardioprotection on myocardial I/R injury through upregulation of mitochondrial fusion and suppression of ROS production.

## 2. Methods

### 2.1. Cell Culture

H9C2 cardiomyocytes were cultured based on a previous study [20]. An in vitro H/R model was applied to mimic myocardial I/R injury. Cells were subcultured at 80% confluence using 0.25% trypsin/ethylenediaminetetraacetic acid [21]. When the cells reached a suitable density, melatonin was then added at a final concentration of 10 mM for 24 hours before H/R injury [22].

### 2.2. Assessment of Cell Viability

A CCK-8 colorimetric experiment was applied determine the viability of H9C2 cells according to a previous study [23]. The cells in each well were subsequently incubated with 10 *μ*L of CCK-8 solution for two hours [24]. Cell viability was determined based on the optical density value, with the average value in control cells being considered as 100% viability [25].

### 2.3. Immunofluorescence Staining

Cells were fixed with 4% v/v paraformaldehyde for 30 min at room temperature and permeabilized with 0.5% v/v Triton X-100 for 10 min [26]. The cells were then washed with PBS and blocked using PBS containing 2% w/v bovine serum albumin and 10% goat serum for 30 min at 37°C [27]. The cells were stained with primary antibodies and visualized with an Alexa Fluor 488–conjugated anti-rabbit secondary antibody (A-11070; Thermo Fisher, Waltham, MA) [28]. The nuclei were stained with DAPI, and images were obtained using a Nikon Eclipse Ti-U fluorescence microscope [29].

RETRACTED

### 2.4. Western Blot Analysis

After SDS-PAGE, protein was transferred from the gels to PVDF membranes using an iBlot system (Invitrogen) [30]. After blocking, the membrane was treated with primary antibodies. After several washes, horseradish peroxidase (HRP) (anti-rabbit IgG, Cat# 7074P2, CST, Danvers, MA; anti87 mouse IgG, Cat# 7076P2, CST) was used [31]. After washing, the signals of blots were detected through ECL reagent (Pierce, Rockford, IL) [32].

### 2.5. qRT-PCR

The RNA was reverse-transcribed into cDNA by transcription Kit [33]. Quantitative PCR was conducted on the Real-Time PCR System (LightCycle480 Instrument II, Roche Diagnostics Inc. Basel, BS, Switzerland) [34]. Total RNA was prepared from mice liver using RNeasy Lipid Tissue Mini Kit (Qiagen) [35]. The relative mRNA expression was normalized to the housekeeper GAPDH levels using the *ΔΔ*CT method.

### 2.6. ELISA

Samples were collected by intracardial punction into BD microtainer tubes. Levels of targeted proteins were analyzed according to manufacturer's instructions (Adiva 1650, Bayer). For the determination of targeted protein levels, 200 mg sample was homogenized in 1 ml 30% KOH at 100°C for 10 min. Samples were left to cool, and 2 ml of ethanol was applied in this study for 24 h at -20°C. The pellet was resuspended in 1 ml 5 N H_2_SO_4_ and incubated for 2 h at 100°C. Finally, samples were neutralized with 1 N NaOH and phenolphthalein (Fluka) as pH indicator.

### 2.7. RNA Silencing

Cells were transfected with indicated siRNA scrambled siRNA (OriGene, Rockville, MD) [36], or siRNA targeting OPA1 (OriGene, Rokville, MD). At 48 hours after transfection, the OPA1 mRNA level was detected by qPCR kit [37].

### 2.8. Statistical Analyses

All data in this study are expressed as the mean ± SD. SPSS software (version 13.0) was used, and the significant differences were analyzed using ANOVA followed by general linear model procedures using a univariate approach. *P* < 0.05 was considered statistically significant.

## 3. Results

### 3.1. Melatonin Activates Mitochondrial Fusion in Hypoxia/Reoxygenation- (H/R-) Treated H9C2 Cells

As shown in Figure 1(a), the transcription of optic atrophy 1 (*OPA1)* was downregulated in H/R-treated H9C2 cardiomyocytes compared with normal cells. We then performed immunofluorescence analyses, which indicated that the OPA1 protein expression was rapidly reduced in cardiomyocytes following H/R injury (Figures 1(b) and 1(c)). Treatment of melatonin induced both the mRNA and protein expression of OPA1 in H/R-treated cardiomyocytes (Figures 1(b) and 1(c)). We then examined the mRNA levels of mitochondrial fusion markers such as mitofusins 1 and 2 (*Mfn1* and *Mfn2*) and found that they were significantly downregulated in H/R-treated H9C2 cardiomyocytes; however, melatonin treatment reversed these effects (Figures 1(d) and 1(e)). These results illustrated that melatonin augmented OPA1-dependent mitochondrial fusion in H/R-treated H9C2 cells.

RETRACTED

### 3.2. Loss of *OPA1* Abolishes Melatonin-Induced Cardioprotection in H9C2 Cells

Next, we evaluated whether melatonin could protect H9C2 cardiomyocytes against H/R injury and whether this protection depended on OPA1-induced mitochondrial fusion. For this purpose, small interfering RNA- (siRNA-) mediated knockout experiment was used. As shown in Figure 2(a), H/R injury repressed the viability of H9C2 cardiomyocytes. Melatonin treatment sustained the viability of H/R-treated cardiomyocytes; however, *OPA1* siRNA abolished this effect (Figure 2(a)). We then assessed caspase-3 activity using an enzyme-linked immunosorbent assay (ELISA), which confirmed that H/R injury induced cardiomyocyte apoptosis (Figure 2(b)). Melatonin inactivated caspase-3 in an OPA1-dependent fashion in H/R-treated cells (Figure 2(b)).

Subsequently, we examined the roles of melatonin in cardiomyocyte structure by using troponin T staining to visualize the cardiomyocyte contraction skeleton. Cardiomyocytes exposed to H/R injury exhibited abnormal cardiomyocyte contraction skeletons or reduced troponin T levels (Figures 2(c) and 2(d)). Melatonin treatment restored the levels of troponin T, while *OPA1* siRNA negated this action (Figures 2(c) and 2(d)).

A reduced cellular troponin T level may indicate that troponin T has been secreted into the bloodstream, where it can upregulate cardiac damage markers. Thus, we used ELISAs to analyze the secretion of myocardial injury biomarkers such as lactate dehydrogenase (LDH), troponin T, and creatine kinase- (CK-) MB into the cell culture media of cardiomyocytes. H/R treatment rapidly increased the secretion of LDH, troponin T, and CK-MB from cardiomyocytes (Figures 2(e)–2(g)). Melatonin treatment reduced the secretion of LDH, troponin T, and CK-MB from H/R-treated cells, and this effect primarily depended on OPA1 (Figures 2(e)–2(g)). These results demonstrated that OPA1 contributed to the cardioprotective effects of melatonin during H/R injury.

### 3.3. OPA1 Activation by Melatonin Inhibits Oxidative Stress in Cardiomyocytes

Oxidative stress is one of the main pathogenic contributors to myocardial I/R injury. Considering the cardioprotective effects of melatonin, we next investigated whether melatonin inhibited oxidative stress in cardiomyocytes by promoting OPA1-dependent mitochondrial fusion. Immunofluorescence analyses indicated that H/R injury elevated mitochondrial ROS production in cardiomyocytes (Figures 3(a) and 3(b)). Melatonin treatment suppressed mitochondrial ROS generation in H/R-treated cardiomyocytes, and this effect depended on OPA1-induced mitochondrial fusion (Figures 3(a) and 3(b)).

RETRACTED

We also analyzed the activity of antioxidative molecules using ELISAs. Superoxide dismutase (SOD), glutathione (GSH), and glutathione peroxidase (GPX) levels were reduced in H/R-treated cardiomyocytes relative to normal cells (Figures 3(c)–3(e)). Melatonin restored the concentrations of SOD, GSH and GPX in H/R-treated cardiomyocytes; however, loss of *OPA1* prevented this restoration (Figures 3(c)–3(e)). These data illustrated that melatonin attenuated oxidative stress in cardiomyocytes by activating OPA1-dependent mitochondrial fusion.

### 3.4. Melatonin Sustains Mitochondrial Function by Inducing OPA1 in Cardiomyocytes

Reduced mitochondrial oxidative stress in cardiomyocytes would be expected to promote mitochondrial function and thus attenuate H/R-induced damage. Therefore, we assessed the effects of melatonin treatment on mitochondrial function in cardiomyocytes. First, we used an ELISA to determine the mPTP opening rate. H/R injury promoted mPTP opening in cardiomyocytes, whereas melatonin inhibited this effect (Figure 4(a)). Loss of *OPA1* prevented melatonin from reducing the mPTP opening rate in H/R-treated cells (Figure 4(a)).

Increased mPTP opening reduces the mitochondrial membrane potential. Staining with the JC-1 probe indicated that H/R injury significantly suppressed the mitochondrial membrane potential in cardiomyocytes (Figure 4(b)). Melatonin restored the mitochondrial potential, but *OPA1* siRNA inhibited this alteration (Figure 4(b)).

A reduced mitochondrial membrane potential induces mitochondria-dependent apoptosis, which is characterized by increased Bax and reduced Bcl-2 expression. Using qRT-PCR, we found that H/R injury increased the *Bax/Bcl-2* ratio in cardiomyocytes (Figures 4(c)–4(e)). Melatonin treatment reversed this increase by activating OPA1 in H/R-treated cells (Figures 4(c)–4(e)). These results confirmed that melatonin sustains the mitochondrial function in cardiomyocytes by inducing OPA1-dependent mitochondrial fusion.

## 4. Discussion

In myocardial I/R, a strong oxidative stress response occurs, which promotes myocardial injury and cardiomyocyte death [38, 39]. Although the use of antioxidant therapy would seem to be a logical method to reduce myocardial I/R injury, this approach has yielded varying results in experimental and clinical studies [40, 41], partly because the tested antioxidants cannot enter cells. In this regard, specific antioxidants targeting mitochondria may be more effective [42, 43].

RETRACTED

In addition to oxidative stress, intracellular calcium overload can occur during acute myocardial ischemia [44, 45]. During myocardial reperfusion, this intracellular calcium overload can become aggravated due to cell membrane rupture, oxidative stress-induced endoplasmic reticulum injury, or mitochondrial reenergization and may be accompanied by mitochondrial calcium overload [46, 47]. The reenergization of mitochondria restores the mitochondrial potential [48, 49]. Several studies have demonstrated that administering drug antagonists of the mitochondrial calcium unidirectional transporter or cell membrane calcium channels can reduce the infarction area by 50% [50, 51]. However, this treatment strategy has not yielded positive results in all experimental studies, and calcium antagonists have not achieved beneficial effects during myocardial reperfusion in clinical studies.

*OPA1* is a nuclear coding gene consisting of 31 exons and spanning 100 kilobases at the end of the human 3q chromosome [52, 53]. Like most genes encoding mitochondrial proteins, *OPA1* is expressed at different levels in various organs. The open reading frame of human *OPA1* generates eight mRNAs [54, 55]. A series of shearing reactions generate long (“L”) and short (“s”) subtypes of OPA1. The *s* subtype promotes mitochondrial network fusion in cooperation with mitofilin (outside the outer membrane) and the *L* subtype (bound to the inner membrane) [56, 57].

OPA1 is important for energy metabolism because it is located in the main site of oxidative phosphorylation [58, 59]. OPA1 prevents proton leakage, promotes the efficient transport of electrons among the respiratory chain complexes, and stabilizes the mitochondrial membrane potential. *OPA1* mutations in fibroblast lines have been found to cause coupling defects in oxidative phosphorylation, and RNA interference of *OPA1* was shown to severely reduce endogenous respiration [60, 61]. OPA1 also links mitochondrial dynamics with apoptosis, as it helps to retain cytochrome C in the ridge space, thereby preventing apoptosis induced by internal stimuli [62, 63]. Accordingly, low expression or pathogenic mutations of *OPA1* have been reported to promote apoptosis.

Previous studies have indicated that plasma melatonin levels are reduced in patients with coronary heart disease [64, 65]. Melatonin and GSH levels were significantly suppressed, and lipid peroxidase levels were elevated in patients with myocardial infarction [66, 67], possibly as a result of substantial consumption of melatonin during the oxidative stress response [68, 69]. In a study of isolated mouse heart retrograde aortic perfusion, melatonin inhibited the opening of the mPTP and mitochondrial cytochrome C activation [70, 71], thus reducing the myocardial infarction area and necrotic injury. Moreover, melatonin also inhibited myocardial apoptosis, maintained the mitochondrial structural stability of ischemic cardiomyocytes, promoted ATP synthesis, and improved cardiac function [72–74].

RETRACTED

Our data found that melatonin induces OPA1-dependent mitochondrial fusion, thus reducing mitochondrial oxidative stress, enhancing mitochondrial function, and improving cardiomyocyte survival during H/R injury. However, this study had several limitations. We only performed cellular experiments to analyze the relationship between melatonin and OPA1-induced mitochondrial fusion; thus, animal studies are needed to validate our reports. In addition, we only tested one concentration of melatonin in cardiomyocytes; so, further research is needed to determine the most effective dose.

## Figures and Tables

**Figure 1:** Melatonin activates OPA1-induced mitochondrial fusion in H/R-treated H9C2 cells. (a) qRT-PCR was used to analyze the transcription of *OPA1* in H9C2 cardiomyocytes subjected to H/R injury and treated with melatonin. (b, c) Western blotting was used to observe the OPA1 expression in H/R-treated H9C2 cardiomyocytes. (d, e) qRT-PCR was used to detect the transcription of *Mfn1* and *Mfn2*. ^∗^*P* < 0.05 vs. control.

**Figure 2:** Loss of *OPA1* abolishes the cardioprotective effects of melatonin in H9C2 cells. (a) Cell viability was determined using a CCK-8 assay. (b) An ELISA was applied to analyze caspase-3 activity. (c, d) An immunofluorescence assay was used to detect troponin T levels in cardiomyocytes following H/R injury and melatonin treatment. (e)–(g) ELISAs were used to measure cardiac damage markers such as LDH, troponin T, and CK-MB. ^∗^*P* < 0.05 vs. control.

**Figure 3:** OPA1 activation by melatonin inhibits oxidative stress in cardiomyocytes. (a, b) Mitochondrial ROS production was measured through immunofluorescence assays. (c)–(e) ELISAs were applied to analyze SOD, GSH, and GPX activity. ^∗^*P* < 0.05 vs. control.

**Figure 4:** Melatonin sustains the mitochondrial function by inducing OPA1 in cardiomyocytes. (a) mPTP opening was analyzed through an ELISA. (b) A JC-1 probe was used to observe changes in the mitochondrial membrane potential. (c)–(e) qRT-PCR was performed to analyze *Bcl-2*, *Bax*, and *Bax/Bcl-2* levels. ^∗^*P* < 0.05 vs. control.

RETRACTED

## Data Availability

The analyzed data sets generated during the present study are available from the corresponding author on reasonable request.
